# Effects of Moxibustion Combined with Ultrashort Wave on Pain and Oxidative Stress in Elderly Patients with Knee Osteoarthritis

**DOI:** 10.1155/2022/3921021

**Published:** 2022-05-09

**Authors:** Yan Wang, Tingquan Yan, Xiaojing Mu, Hong Dong, Jinman Su

**Affiliations:** ^1^First Outpatient Department, 971st Hospital, People's Liberation Army Navy, Qingdao, Shandong 266071, China; ^2^Ten Branches of Recuperation, Navy Qingdao Special Service Convalescent Center, Qingdao, Shandong 266071, China

## Abstract

**Objective:**

To explore the effect of moxibustion instrument combined with ultrashort wave on pain and oxidative stress in elderly patients with knee osteoarthritis (KOA).

**Method:**

84 elderly patients with knee osteoarthritis treated in our hospital from May 2020 to June 2021 were randomly divided into observation group (*n* = 42) and control group (*n* = 42). The observation group was treated with moxibustion instrument combined with ultrashort wave, while the control group was treated with moxibustion instrument. The clinical efficacy of the two groups was compared, and the pain of the two groups was evaluated by visual analogue scale (VAS). Lysholm knee joint score scale and osteoarthritis index (WOMAC) scale of Western Ontario and McMaster University were used to evaluate the knee joint function of the two groups, and the levels of interleukin-1*β* (IL-1*β*), tumor necrosis factor *α* (TNF-*α*), serum superoxide dismutase (SOD), serum malondialdehyde (MDA), serum miR-155, and NLRP3 were detected in the two groups, and the comprehensive quality of life assessment questionnaire-74 was used, and the adverse reactions were compared between the two groups.

**Results:**

The total effective rate of observation group (90.48%) was higher than that of control group (69.05%) (*P* < 0.05). After treatment, VAS, Lysholm knee joint, WOMAC, quality of life scores, IL-1*β*, TNF-*α*, SOD, MDA, miR-155, and NLRP3 in the observation group were better than those in the control group, and the differences were statistically significant (*P* < 0.05). There were no obvious adverse reactions in both groups*. Conclusion*. Moxibustion instrument combined with ultrashort wave can effectively improve knee joint pain, knee joint function, inflammatory reaction, oxidative stress reaction, and quality of life in elderly KOA patients, and the therapeutic effect is good.

## 1. Introduction

Knee osteoarthritis (KOA), also known as degenerative knee osteoarthritis, is a chronic inflammatory joint disease. Its main clinical features are degeneration, destruction and hyperosteogeny of articular cartilage, which will lead to pain and impaired joint function [1]. The incidence of KOA among the elderly over 65 years old in China has reached 85%, and the pathogenesis of KOA is still unclear. According to relevant studies, inflammation and oxidative stress are closely related to the occurrence and development of KOA [2]. Moxibustion has been widely used in the treatment of KOA. Moxibustion can effectively relieve the clinical symptoms of patients. In addition, as a common treatment of traditional Chinese medicine, moxibustion has been proved to effectively regulate the function of viscera and improve the immunity and circulation of the body [3, 4]. The moxa smoke produced by traditional moxibustion greatly irritates the eyes and nose. The new moxibustion instrument puts moxa wool under the heating element moxibustion head, fixes the moxibustion head on the acupoints, and lights the moxibustion head to raise the moxa wool temperature, thus, stimulating the skin acupoints to play a therapeutic role and avoiding the shortcomings of traditional moxibustion. Ultrashort wave has strong penetrating power and warming effect, which can be applied locally by alternating magnetic field, play the role of dilating blood vessels and accelerating blood flow, help to eliminate local edema, relieve pain, and improve local nutrition and metabolism. In addition, ultrashort wave can also improve venous stasis, relieve the destruction of bone joints by intraosseous high pressure, delay the process of osteoarthritis, promote local blood circulation, accelerate metabolism, fully nourish local blood vessels, nerves, and muscles, and play the role of expelling cold and dehumidifying. At present, the randomized clinical research of moxibustion instrument combined with ultrashort wave therapy is still lacking, and it has been clinically used. The purpose of this study is to explore the effect of moxibustion instrument combined with ultrashort wave therapy on pain and oxidative stress of KOA patients. It provides clinical guidance significance for the application of moxibustion instrument combined with ultrashort wave therapy.

## 2. Materials and Methods

### 2.1. General Information

A total of 84 elderly patients with knee osteoarthritis who were admitted to our hospital from May 2020 to June 2021 were randomly divided into observation group and control group. There are 42 patients in each group. There were 12 males and 30 females in the observation group; the age ranged from 60 to 77 years, with an average of (67.67 ± 4.46) years; the course of disease ranged from 3 months to 11 years, with an average of (6.04 ± 2.60) years. There were 16 males and 26 females in the control group; the average age was (67.07 ± 4.04) years; the course of disease ranged from 5 months to 19 years, with an average of (6.06 ± 2.56) years. There was no statistical difference between the above base data of the two groups of patients (*P* > 0.05), and they were comparable. This study was approved by the hospital ethics committee.

### 2.2. Diagnostic Criteria

Diagnostic criteria of western medicine: knee osteoarthritis was diagnosed according to “Guidelines for Diagnosis and Treatment of Osteoarthritis” [5]: ① repeated pain of knee joint in the past month; ② X-ray film in standing or weight-bearing position showed that the joint space was narrowed, subchondral bone sclerosis, joint margin, and cystic degeneration were formed; ③ arthritis at least twice was cool and sticky, and the white blood cell count was less than 2000/ml; ④ morning stiffness ≤3 min; ⑤ there is bone friction during activities. If ①+② or ①+③+④+⑤ is satisfied, KOA can be diagnosed. Standard of syndrome differentiation of traditional Chinese medicine: refer to the diagnosis and treatment plan of knee arthritis (knee osteoarthritis) [6]. ① Wind-cold-dampness arthralgia syndrome is characterized by soreness and pain in limb joints, fixed pain, feeling of knife cutting or obvious severe pain, or obvious swelling in the affected part, inability of joints to move flexibly, fear of wind-cold, feeling comfortable when getting hot, pale tongue with white fur and tight pulse. ② Rheumatic rheumatism is characterized by acute onset, red and swollen joints, pain, cold, and comfortable, accompanied by general fever, erythema of skin, red tongue and yellow fur, and slippery pulse. ③ Congestion arthralgia syndrome limb tingling, fixed pain, local stiffness, numbness, and purple tongue with white and dry fur. ④ Patients with deficiency of liver and kidney have dull pain in knee joint, soreness and pain in waist and knees, aggravation of fatigue, less red tongue coating, and deep and thin pulse.

### 2.3. Including and Exclusion Criteria

Inclusion criteria: ① patients who all meet the diagnostic criteria of arthritis and TCM syndrome differentiation criteria in the guide to diagnosis and treatment of osteoarthritis [5]; ② the diagnosis of knee osteoarthritis by imaging examination; ③ age ≥ 60 years old; ④ all patients voluntarily participated in this study and signed informed consent forms. Exclusion criteria: ① knee pain caused by other diseases; ② severe deformation of knee joint structure; ③ those who received acupuncture or ultrashort wave therapy 3 months before admission; ④ patients with severe mental illness; ⑤ patients with suppurative infection; ⑥ those who are treated with other drugs (such as nonsteroidal anti-inflammatory drugs, chondroprotective agents, and adrenal cortex hormones).

### 2.4. Methods

The control group was treated with ultrashort wave, using Shanghai TC1 ultrashort wave therapeutic apparatus with 200 w output power. One electrode was placed under the knee joint, the other electrode was placed above the knee joint, and the two electrodes were placed in parallel. The heat was set at 100~120 mA, 20 minutes/time, the treatment frequency was once a day, with 10 times as a course of treatment, and each course interval was 3 ~ 5 days. The observation group was treated with moxibustion instrument combined with ultrashort wave. Ultrashort wave treatment is the same as that of the control group. Moxibustion instrument treatment: the patient takes a sitting position, the knee joint of the affected side flexes at an angle of 90 degrees, and the needle is inserted vertically from the blood sea and Liang Qiu with a depth of 1-1.5 inches. The inner and outer knee eyes use a 3-inch millineedle, and the needle tip penetrates into the center of the knee joint for 2-2.5 inches. After getting angry, twist, with the degree of soreness felt in the deep part of the knee joint, leave the needle and place the moxibustion head of moxibustion instrument in it, and pass the moxa bag, then, four moxibustion instrument heads are passed through the needle handle from the warm needle hole and placed on the moxa pad. The moxibustion heads are fixed with 1 cm × 20 cm long footsteps and cross-fixed. After leaving for 30 min minutes, twist the needle handle twice, remove the footsteps when taking out the needle, moxibustion the head, and then take out the needle. The moxibustion instrument is treated once a day, and every 10 days is a course of treatment. Both groups were evaluated after one course of treatment [6].

### 2.5. Observation Index

① Clinical efficacy. ② Pain situation: Visual Analogue Scale (VAS) [7] was used to evaluate the pain of patients before and after treatment. On the 10 cm long line engraved with numbers in the center of the card, there was a sliding cursor with scores of 0 ~ 10 at both ends, representing “painless” to “the most severe pain.” ③ Knee joint function before and after treatment, Lysholm Knee Joint Scoring Scale [8] was used to evaluate the knee joint function of the two groups. The scoring standard indexes included limping (5 points), supporting (5 points), squatting (5 points), climbing stairs (10 points), swelling (10 points), locking (15 points), stability (25 points), and pain (25 points), total score: 0 ~100. ④ The Western Ontario and McMaster University Osteoarthritis Index (WOMAC) scale [9] was used to evaluate the knee joint function of the two groups before and after treatment. The scale included pain, stiffness, and joint function, with a total score of 0 ~ 96. The higher the score, the more serious the illness. ⑤ Inflammatory factor level before and after treatment, 5 ml of fasting venous blood was taken from patients, and the upper serum was separated by centrifugation at room temperature at 3000 r/min for 15 min. The levels of interleukin-1*β* (IL-1*β*) and *α* (tumor necrosis factor *α* (TNF-*α*)) were determined by enzyme-linked immunosorbent assay. ⑥ Oxidative stress index level takes the abovementioned serum to be tested, the serum superoxide dismutase (SOD) level is determined by enzyme-linked immunosorbent assay, and the serum malondialdehyde (MDA) level is determined by double antibody sandwich assay. ⑦ Serum miR-155 and NLRP-3 levels. The expression levels of miR-155 and NLRP-3 in the two groups were measured by qRT-PCR method [10]. Take the abovementioned serum to be measured, extract the total RNA from the serum with Trizol reagent, precipitate and concentrate it with isopropanol, then wash it with 75% alcohol, add 100 *μ*l of diethyl pyrocarbonate (DEPC) water after drying, and detect the purity and integrity of the obtained RNA. RNA was reverse transcribed intocRNA, which was stored at -20°C. The total reaction system was 25 *μ*l, including 9 ml SYBR Green Mix 9 *μ*l, and RNase-free water was used to make up 25 *μ*l. U6 was used as the internal reference of miR-155, and the reaction program was set at 95°C for 20 s, 95°C for 10 s, 60°C for 20 s, and 70°C for 10 s, totally 40 cycles. The internal reference of NLRP3 is *β*-actin, and the reaction conditions are set at 95°C for 95°C 5 min, 95°C for 30 s, 55°C for 30 s, and 72°C for 1 min. There are 35 cycles in total. U6ispositive: CTTAGTTGCATGCAG, and reverse: AATCCTGTATAAGTC; miR-155 forward: GTCCCAATGCTGTCT, reverse GGAAGTTGCATGCAT; B-actin forward: GTAGTTTCGTGGATGCCACAG, reverse: GAGCTACGAGCTGCCTGACG; NLRP3 forward: CCCCGTGAGTCCCATTA, reverse GACGCCCAGTCCACAT. The miR-155 and NLRP3 levels were calculated by 2-△△Ct method. ⑧ The quality of life before and after treatment was evaluated by the comprehensive quality of life assessment questionnaire-74 (GQOLI-74) [11], which included four dimensions, four factors in each dimension, and a total of 16 factors (64 items). The highest score of each factor was 20 points, and the highest score of each dimension was 80 points. The higher the score, the better the quality of life. ⑨ Adverse reactions (skin pruritus, increased intermittent needle-like pain in the knee joint, infection, etc.).

### 2.6. Evaluation Standard of Curative Effect

The criteria for evaluating the treatment effect of the two groups of patients are as follow: cure: joint pain, swelling, and pain disappeared, and activity function returned to normal, Lysholm knee joint score was 80~100; improvement: joint pain and swelling were reduced, and function was improved. Lysholm knee joint score was 60~79; unhealed: no change in joint pain and swelling, Lysholm knee joint score < 60. Total effective = cure + improvement.

### 2.7. Statistical Method

SPSS 20.0 statistical software was used to analyze and process the data. The measurement data were expressed as (*x* ± *s*). Independent sample *t*-test was performed for the comparison between groups. Paired *t*-test was used for the comparison before and after treatment. The counting data were expressed as frequency and constituent ratio, and *χ*^2^ test was performed. *P* < 0.05, indicating that the difference was statistically significant.

## 3. Result

### 3.1. Comparison of the Clinical Efficacy between the Two Groups

The total effective rate of observation group was 90.48%, while that of control group was 69.05%, and the difference was statistically significant (*P* < 0.05), see Table 1.

### 3.2. Comparison of the VAS Score and the WOMAC Score between the Two Groups

Before treatment, there was no significant difference in VAS score, Lysholm knee joint score, and WOMAC score between the two groups (*P* > 0.05). After treatment, the VAS score and WOMAC score of the two groups decreased significantly, while Lysholm knee joint score increased significantly. The improvement degree of each score in the observation group was greater than that in the control group, and the difference was statistically significant (*P* < 0.05), see Table 2.

### 3.3. Comparison of Inflammatory Response Indexes between Two Groups

Before treatment, there was no significant difference in IL-1*β* and TNF-*α* levels between the two groups (*P* > 0.05). After treatment, the levels of IL-1*β* and TNF-*α* in both groups decreased significantly, and the observation group was lower than the control group, with a statistically significant difference (*P* < 0.05), see Table 3.

### 3.4. Comparison of Oxidative Stress Reaction Indexes between Two Groups

Before treatment, there was no significant difference in SOD and MDA levels between the two groups (*P* > 0.05). After treatment, SOD level increased significantly, and MDA level decreased significantly in the two groups. The improvement degree of each index in the observation group was greater than that in the control group, and the difference was statistically significant (*P* < 0.05), see Table 4.

### 3.5. Comparison of miR-155 and NLRP3 Levels between Two Groups

Before treatment, there was no significant difference in the levels of miR-155 and NLRP3 between the two groups (*P* > 0.05). After treatment, the level of miR-155 decreased and the level of NLRP3-3 increased in the two groups. The improvement degree of each index in the observation group was greater than that in the control group, and the difference was statistically significant (*P* < 0.05), see Table 5.

### 3.6. GQOLI-74 Score of Life between Two Groups

Before treatment, there was no significant difference in the scores of physical function, psychological function, social function, and material life function between the two groups (*P* > 0.05). After treatment, the scores of physical function, psychological function, social function, and material life function in the two groups all increased, and the improvement degree of each score in the observation group was greater than that in the control group, with statistical significance (*P* < 0.05), see Table 6.

### 3.7. Adverse Effect

No obvious adverse reactions occurred in both groups (*P* > 0.05).

## 4. Discuss

Ultrashort wave is a kind of high-frequency electromagnetic wave, which can uniformly heat the surface and deep tissues of the body and can effectively relieve the chronic inflammatory reaction of fat, bone in muscle, synovium, joint capsule, and other structures of joints. By inhibiting sensory nerve, relieving muscle spasm, and improving blood circulation, it can effectively promote metabolism and excretion of pain-causing substances, relieve various body pains, dilate blood vessels, accelerate blood and lymph circulation, enhance blood vessel permeability, enhance leukocyte phagocytosis, adjust the pH of the focus area to make it alkaline, reduce tissue acidosis, and play the roles of eliminating inflammatory reaction, relieving pain, and restoring motor function. Knee osteoarthritis belongs to the category of “bone arthralgia” in traditional Chinese medicine. The disease is mostly caused by wind, cold, and dampness blocking meridians, which can lead to the unsmooth movement of qi and blood, and the stagnation of qi and blood causes pain. When arthralgia is cold and wet, qi and blood are not smooth, which can lead to aggravation of symptoms; when it is hot, it can smooth meridians, smooth qi and blood and relieve symptoms. The heat of moxibustion fire has the effect of activating qi and blood circulation and enhancing patients' disease resistance. Traditional moxibustion needs to replace moxa velvet several times during treatment. If moxa velvet falls carelessly, it may burn patients. The whole process needs to be paid close attention, which will seriously affect the work efficiency of medical staff. Moxibustion instrument has improved the traditional moxibustion method. On the basis of ensuring the therapeutic effect, there is no need to worry that moxa velvet will burn patients, and it can treat many patients at the same time, which greatly improves the working efficiency of medical staff. In this study, traditional Chinese medicine therapy and physical therapy were combined. The results showed that the total effective rate of the observation group (90.48%) was significantly higher than that of the control group (69.05%). After treatment, the improvement degree of VAS score, WOMAC score, Lysholm knee joint score, and GQOLI-74 score in the observation group was significantly higher than that in the control group, indicating that moxibustion combined with ultrashort wave can effectively improve the pain and knee joint function of patients, and the treatment effect is good, which may be because moxibustion in the observation group has further played the role of regulating qi and blood, relieving pain and improving joint function on the basis of ultrashort wave treatment. In the study of Li Xiaojuan et al. [12], the effect of warm acupuncture combined with ultrashort wave in treating knee arthritis is better than that of ultrashort wave alone, and the results of this study are similar.

Comparison of inflammatory response between the two groups, according to related studies, the serum levels of IL-1*β* and TNF-*α* in KOA patients are higher than those in healthy people [13, 14]. Excessive levels of inflammatory factors can lead to abnormal cartilage metabolism in knee osteoarthritis, lead to articular cartilage deformation, and destroy the normal structure of knee joint. IL-1*β* and TNF-*α* can promote the degradation of extracellular matrix, damage cartilage, promote the proliferation and differentiation of synovial fibroblasts, destroy articular cartilage and bone, and induce the production of inflammatory mediators, further aggravating the patient's condition. In this study, after treatment, the levels of IL-1*β* and TNF-*α* in the observation group were lower than those in the control group, indicating that moxibustion combined with ultrasound can effectively improve the inflammatory response of KOA patients, which may be related to the anti-inflammatory effect of moxibustion. According to research, miR-155 is closely related to KOA inflammation, which can lead to stem cell depletion [15]. The expression of miR-155 in synovial fluid of KOA patients is more than twice as high as that of healthy people, which may be related to the pathogenesis of KOA [16]. Estradiol can further inhibit the activation of NLRP3 inflammasome by reducing the levels of NLRP3 mRNA and protein through estrogen receptor *β*. Studies have suggested that NLRP3 is in a low level in KOA process, which may play a protective role in the process of inflammatory stress [17, 18]. miR-155 can promote the secretion of TNF-*α*, and NLRP3-3 inflammatory corpuscles can inhibit the expression of TNF-*α*, thus playing a protective role. In this study, after treatment, the level of miR-155 decreased, the level of NLRP-3 increased in the observation group, and the improvement degree of each index was greater than that in the control group, indicating that moxibustion combined with ultrashort wave can effectively regulate the levels of miR-155 and NLRP-3, and the expression levels of miR-155 and NLRP-3 are closely related to the levels of inflammatory factors. Ultrashort wave can promote metabolism and eliminate inflammation. Previous studies have shown that moxibustion can effectively improve the inflammatory response of KOA patients, and the combination therapy can effectively improve the expression of miR-155 and NLRP3-3 by playing the role of multitarget therapy. The quality of life of the two groups is compared.

Oxygen-free radicals produced by oxidative stress can play an important role in the pathogenesis of KOA. Under normal circumstances, the generation of oxygen free radicals keeps a dynamic balance, and the increase of oxygen free radicals in KOA patients can lead to chondrocyte death and cartilage damage. According to research, SOD level is negatively correlated with KOA disease severity, while MDA level is positively correlated with disease severity [19]. In this study, after treatment, the SOD level in the observation group increased significantly, MDA level decreased significantly, and the improvement degree of each index was greater than that in the control group, which indicated that moxibustion combined with ultrasound could effectively improve the oxidative stress reaction of KOA patients, possibly because moxibustion could effectively reduce the level of oxygen free radicals in serum of KOA patients, and its specific mechanism needs to be further explored. Previous studies have shown that moxibustion can effectively improve the oxidative stress level of KOA patients [20, 21], and the results of this study are consistent with it.

To sum up, moxibustion instrument combined with ultrashort wave can effectively improve the pain and function of knee joint of elderly KOA patients, effectively relieve their inflammatory reaction and oxidative stress reaction, and improve their quality of life, which has clinical application value.

## Figures and Tables

**Table 1:** Comparison of clinical efficacy between two groups (*n*(%)).

Groups	Cure	Improve	Ineffective	Effective
Observation group (*n* = 42)	11 (26.19)	27 (64.29)	4 (9.52)	38 (90.48)
Control group (*n* = 42)	6 (14.29)	23 (54.76)	13 (30.95)	29 (69.05)
*χ* ^2^ value				5.974
*P* value				0.015

**Table 2:** Comparison of the VAS score and the WOMAC score between the two groups (^−^*x* ± *s*, points).

Groups	VAS score		Lysholm knee joint score		WOMAC score	
	Before treatment	After treatment	Before treatment	After treatment	Before treatment	After treatment
Observation group (*n* = 42)	6.21 ± 0.65	2.67 ± 0.82^a^	42.00 ± 4.52	75.76 ± 6.10^a^	29.26 ± 2.65	14.83 ± 1.71^a^
Control group (*n* = 42)	6.48 ± 0.80	3.88 ± 1.33^a^	40.80 ± 4.93	67.29 ± 5.58^a^	29.07 ± 2.31	23.86 ± 2.35^a^
*T* value	1.647	5.046	1.153	6.645	0.351	20.103
*P* value	0.103	<0.001	0.252	<0.001	0.726	<0.001

Note: compared with the same group before treatment, ^a^*P* < 0.05.

**Table 3:** Comparison of inflammatory response indexes between two groups (^−^*x* ± *s*).

Groups	IL-1*β* (ng/L)		TNF-*α* (ng/L)	
	Before treatment	After treatment	Before treatment	After treatment
Observation group (*n* = 42)	38.26 ± 3.83	22.96 ± 1.82^a^	88.65 ± 10.26	51.13 ± 5.09^a^
Control group (*n* = 42)	37.77 ± 3.15	27.33 ± 2.58^a^	87.74 ± 9.04	56.66 ± 5.08^a^
*T* value	0.637	8.962	0.435	4.986
*P* value	0.526	<0.001	0.665	<0.001

Note: compared with the same group before treatment, ^a^*P* < 0.05.

**Table 4:** Comparison of oxidative stress reaction indexes between two groups (^−^*x* ± *s*).

Groups	SOD (NU/mL)		MDA (nmol/L)	
	Before treatment	After treatment	Before treatment	After treatment
Observation group (*n* = 42)	6.18 ± 1.52	11.10 ± 1.10^a^	8.43 ± 1.07	5.50 ± 1.19^a^
Control group (*n* = 42)	6.07 ± 1.22	9.22 ± 1.52^a^	8.80 ± 1.12	6.98 ± 1.25^a^
*T* value	0.378	6.485	1.558	5.530
*Pvalue*	0.706	<0.001	0.123	<0.001

Note: compared with the same group before treatment, ^a^*P* < 0.05.

**Table 5:** Comparison of miR-155 and NLRP3 levels between two groups (^−^*x* ± *s*).

Groups	miR-155		NLRP3	
	Before treatment	After treatment	Before treatment	After treatment
Observation group (*n* = 42)	3.82 ± 1.16	1.85 ± 0.60^a^	52.20 ± 5.44	81.48 ± 8.29^a^
Control group (*n* = 42)	4.03 ± 1.42	2.23 ± 0.71^a^	52.55 ± 5.73	70.14 ± 7.02^a^
*T* value	0.731	4.619	0.291	6.764
*P* value	0.467	<0.001	0.772	<0.001

Note: compared with the same group before treatment, ^a^*P* < 0.05.

**Table 6:** GQOLI-74 score between two groups (^−^*x* ± *s*).

Groups	Somatic function		Psychological function		Social function		Material life function	
	Before treatment	After treatment	Before treatment	After treatment	Before treatment	After treatment	Before treatment	After treatment
Observation group (*n* = 42)	44.29 ± 3.78	70.67 ± 5.51^a^	46.62 ± 4.13	70.19 ± 6.92^a^	46.79 ± 4.38	65.60 ± 6.30^a^	49.43 ± 5.38	72.81 ± 4.81^a^
Control group (*n* = 42)	44.62 ± 6.79	57.64 ± 4.67^a^	46.38 ± 4.15	58.79 ± 5.04^a^	47.10 ± 3.21	59.26 ± 5.51^a^	49.52 ± 5.45	61.67 ± 6.89^a^
*T* value	0.278	11.691	1.419	8.633	0.369	4.904	0.081	8.590
*P* value	0.782	<0.001	0.160	<0.001	0.713	<0.001	0.936	<0.001

Note: compared with the same group before treatment, ^a^*P* < 0.05.

## Data Availability

The labeled dataset used to support the findings of this study are available from the corresponding author upon request.

## References

[1] Kan H. S., Chan P. K., Chiu K. Y. (2019). Non-surgical treatment of knee osteoarthritis. *Hong Kong Medical Journal*.

[2] Scanzello C. R. (2017). Role of low-grade inflammation in osteoarthritis. *Current Opinion in Rheumatology*.

[3] Wang X., Jiang Y., Xiong J. (2020). Moxibustion for treating knee osteoarthritis. *Medicine (Baltimore)*.

[4] Jian-Hui S., Hai-Ru H., Xiao-Qin L. I., Hong-Mei L. I., Li-Ping K., Yuan Z. (2020). Comparison of therapeutic effect of moxibustion materials from different places and storage periods on knee osteoarthritis. *Zhongguo Zhong Yao Za Zhi*.

[5] Oste (2007). *Branch of Chinese Medical Association*.

[6] LiShumei W. Z., Shuhua C. (2020). Observation and nursing of the effect of grain moxibustion combined with ultrashort wave in the treatment of degenerative knee arthritis. *Contemporary Nurse: First Issue*.

[7] Bing S., Xiaoming C. (2012). Visual simulation scoring method VAS. *Journal of Neurosurgery*.

[8] Kocher M. S., Steadman J. R., Briggs K. K., Sterett W. I., Hawkins R. J. (2004). Reliability, validity, and responsiveness of the Lysholm knee scale for various chondral disorders of the knee. *The Journal of Bone and Joint Surgery. American*.

[9] Roos E. M., Klässbo M., Lohmander L. S. (1999). WOMAC osteoarthritis index. Reliability, validity, and responsiveness in patients with arthroscopically assessed osteoarthritis. Western Ontario and MacMaster universities. *Scandinavian Journal of Rheumatology*.

[10] Fu W. J., Guo Y. K., Chen H. (2020). Correlation analysis of NLRP3 content and inflammation and oxidative stress in joint synovial tissue of patients with primary osteoarthritis. *Advances in Modern Biomedicine*.

[11] Shen W., Liu X., Zhou A. (2021). Analysis of continuous nursing intervention on aplastic anemia patients based on the information-motivation-behavioral skills model. *Evidence-based Complementary and Alternative Medicine*.

[12] LiXiaojuan T., Wen Y. (2011). Clinical observation of acupuncture and ultra-short wave treatment of knee osteoarthritis. *Liaoning Journal of Traditional Chinese Medicine*.

[13] Liu C. X., Gao G., Qin X. Q., Deng C. Q., Shen X. J. (2020). Correlation analysis of C-terminal telopeptide of collagen type II and interleukin-1*β* for early diagnosis of knee osteoarthritis. *Orthopaedic Surgery*.

[14] Yıldız K., Boy F. (2021). Serum progranulin to TNF-*α* ratio in patients with gonarthrosis. *Acta Orthopaedica et Traumatologica Turcica*.

[15] Li G. S., Cui L., Wang G. D. (2021). miR-155-5p regulates macrophage M1 polarization and apoptosis in the synovial fluid of patients with knee osteoarthritis. *Experimental and Therapeutic Medicine*.

[16] Li S. H., Wu Q. F. (2021). MicroRNAs target on cartilage extracellular matrix degradation of knee osteoarthritis. *European Review for Medical and Pharmacological Sciences*.

[17] Zhao L. R., Xing R. L., Wang P. M. (2018). NLRP1 and NLRP3 inflammasomes mediate LPS/ATP-induced pyroptosis in knee osteoarthritis. *Molecular Medicine Reports*.

[18] Xiao Y., Ding L., Yin S. (2020). Relationship between the pyroptosis of fibroblast-like synoviocytes and HMGB1 secretion in knee osteoarthritis. *Molecular Medicine Reports*.

[19] Chen Y., Wang R. Q., Liu J. X. (2020). Effect of moxibustion on inflammatory factors and oxidative stress factors in patients with knee osteoarthritis: a randomized controlled trial. *Zhongguo Zhen Jiu*.

[20] Xu H., Zhao H., Kang L. (2018). Moxibustion using different habitat moxa floss for moderate to severe primary knee osteoarthritis: study protocol for a three-armed randomized, double-blinded, sham-controlled trial. *Trials*.

[21] Chen Y., Jia Y. J., Jh L. (2020). Comparision of therapertic effect of different acupuncture methods for knee osteoarthritis. *Zhen Ci Yan Jiu*.

